# Network Pharmacology and In Vivo Analysis of Dahuang-Huangqi Decoction Effectiveness in Alleviating Renal Interstitial Fibrosis

**DOI:** 10.1155/2022/4194827

**Published:** 2022-05-25

**Authors:** Yan Luo, Chen Xuan, Junxiong Cheng, Yu Xiong, Wenfu Cao

**Affiliations:** ^1^College of Traditional Chinese Medicine, Chongqing Medical University, Department of Chinese Traditional Medicine, The First Affiliated Hospital of Chongqing Medical University, No. 1 Yixueyuan Road, Yuzhong District, Chongqing 400016, China; ^2^Chongqing Key Laboratory of Traditional Chinese Medicine for Prevention and Cure of Metabolic Diseases, Department of Chinese Traditional Medicine, The First Affiliated Hospital of Chongqing Medical University, No. 1 Yixueyuan Road, Yuzhong District, Chongqing 400016, China; ^3^Chongqing Traditional Chinese Medicine Hospital, No. 6 Panxi Seventh Branch Road, Jiangbei District, Chongqing 400021, China

## Abstract

Dahuang and Huangqi are the most frequently prescribed treatment methods for chronic kidney disease in China. Our study aimed to clarify the pharmacological mechanism of action of Dahuang-Huangqi decoction (DHHQD) in renal interstitial fibrosis (RIF). The intersection of genes targeted by DHHQD active ingredients and RIF target genes was searched using network pharmacology to build a chemical ingredient and disease target network. For *in vivo* analysis, Sprague–Dawley rats with unilateral urethral obstruction (UUO) were administered DHHQD, and their kidney function-related indicators and pathological indices were determined. The expression of core targets was quantified using real-time polymerase chain reaction and western blotting. A total of 139 common targets for DHHQD and RIF in chronic kidney disease were detected. Compared with the untreated UUO rats, the DHHQD-treated rats showed reductions in the following: blood urea nitrogen and serum creatinine levels, kidney tubular atrophy and necrosis, interstitial fibrosis, hyperplasia and abnormal deposition of extracellular matrix, and microstructural changes in the mesangial matrix and glomerular basement membrane. DHHQD treatment significantly regulated the levels of renal core proteins, such as eNOS, IL-6, EGFR, and VEGF and reduced the mRNA and protein expression of the core targets involved in inflammation pathways, such as PI3K/AKT and TLR4/NF-*κ*B. DHHQD treatment ameliorated the severity of RIF by potentially regulating the AKT/PI3K and TLR4/NF-*κ*B signaling pathways. Our study findings provide insights into the mechanisms associated with DHHQD action and essential data for future research.

## 1. Introduction

Chronic kidney disease (CKD) is currently a prominent global health challenge [1], with a global incidence of approximately 10%–15% [2]. The prevention and treatment of CKD and its related diseases pose an immense challenge to the global health system. Renal interstitial fibrosis (RIF) is a common pathway and pathological feature of CKD progression to end-stage renal disease, which has a complex etiology, a long course, and a severity closely linked to the degree of renal function decline. As the final manifestation of end-stage renal disease, RIF is of great significance for the prevention and treatment of CKD [3]. Therefore, it is important to determine the mechanism of RIF progression to delay the pathological process of CKD and preserve renal function [4].

Traditional Chinese medicine (TCM) maintains that after a long illness, blood stasis is inevitable. In his book “Correcting the Errors in The Forest of Medicine,” Wang Qingren [5] referred to the deficiency of viscera and vital energy, Qi, blood, Yin, and Yang, along with dampness, heat, and blood stasis as the main factors affecting the pathogenesis of CKD. He recommended activation of blood movement and removal of blood stasis, dampness, and turbidity as the main therapeutic approaches.

Data mining of more than 70 popular TCM prescriptions for CKD patients in China revealed that Dahuang (*Rheum palmatum* L., root and rhizome, raw. RL) and Huangqi (*Astragalus membranaceus (Fisch.) Bge.*, root, raw. AM) were the most frequently prescribed treatments [6]. The Herbal Classic of Sheng Nong (Shen Nong Ben Cao Jing, pinyin in Chinese), an ancient Chinese medical text, describes Dahuang as a defecation-promoting, bitter and cold, and purgative medicine. Its efficacy is consistent with the treatment required for CKD. Dahuang is widely used in TCM as an indispensable and specific treatment for curing CKD stages 1–5 and shows good curative effects. In China, Dahuang-based decoctions and other proprietary Chinese medicines have been used to alleviate CKD [7]. Clinical research has demonstrated that Dahuang-based decoctions can improve the symptoms of uremia, reduce the levels of uremic toxins in the blood, and regulate intestinal flora imbalance [7]. Dahuang can also delay the stage wherein hemodialysis is needed. Huangqi is the most important Chinese herb used for Qi supplementation [8]. It is sweet and mildly warm; it supplements Qi, raises yang, boosts Wei Qi to consolidate the exterior, prompts urination to relieve edema, and removes toxins to engender freshness [9]. Huangqi particles have been especially used in Chinese patent medicine for Qi replenishment and as diuretics. Studies have demonstrated that the chemical extract of Huangqi can have antifibrotic and anti-inflammatory effects and may regulate immunity [10]. *Astragalus* polysaccharide can enhance cell proliferation and inhibit megakaryocyte apoptosis [8, 9]. Astragaloside IV, a saponin observed in Huangqi, can modulate inflammation in nephropathic fibrosis [11]. Thus, the herb tonic and laxatives Dahuang and Huangqi are used together when treating renal disorders.

Recent studies have demonstrated that the Dahuang-Huangqi decoction (DHHQD) can reduce urinary protein, serum creatinine (SCr), and blood urea nitrogen (BUN) levels to mitigate renal pathological changes, protect renal function, and delay renal failure. The DHHQD is also used for the treatment of CKD, and its effects have been verified pharmacologically. Specifically, administration of DH and HQ is reportedly associated with lower risks of end-stage renal disease and death among advanced CKD patients [12]. Additionally, DH- and HQ-based decoctions can improve renal inflammatory damage and oxidative stress and inhibit renal fibrosis [7].

Network pharmacology can be used to analyze traditional Chinese formulas in TCM using multiple databases [13] to detect their chemical components, screen their potential active components, predict their targets in related diseases, and explore the underlying therapeutic mechanisms. Network pharmacology can construct the “chemical compositions-active components targets-disease targets-protein interaction (PPI) network” of a traditional Chinese formula [14]. Therefore, it can accelerate the research and development of traditional Chinese herbs and their decoctions.

In this study, we analyzed (i) the effectiveness and mechanism underlying DHHQD action in RIF treatment and (ii) the potential chemically active components and key signaling pathways of DHHQD in RIF.

## 2. Materials and Methods

### 2.1. Preparation of DHHQD

DHHQD is a widely used TCM prescription and consists of the Dahuang *Rheum officinale Baill.,* root and rhizome, raw. RL and Huangqi (*Astragalus membranaceus* (Fisch.) Bge., root, raw. AM) herbs in a 1 : 1 ratio. All herbs were purchased from Chongqing Traditional Chinese Medicine Hospital. The herbs were extracted twice using distilled water and concentrated to 1 g/mL.

### 2.2. Ultra-High Performance Liquid Chromatography-Tandem Mass Spectrometry (UHPLC-MS/MS) Analysis

A 400 *μ*L aliquot of the DHHQD supernatant was passed through a 0.22 *μ*m filter membrane and subsequently transferred to an autosampler vial for UHPLC-MS/MS analysis. LC-MS/MS analysis was performed on an Agilent ultra-high performance liquid chromatography 1290 UPLC system with a Waters UPLC BEH C18 column (1.7 *μ*m; 2.1 × 100 mm). The following conditions were applied: column temperature, 55°C; sample injection volume, 5 *μ*L; flow rate, 0.5 mL/min; and mobile phase, 0.1% formic acid in water (A) and 0.1% formic acid in acetonitrile (B). A multistep linear elution gradient program was implemented as follows: 0–11 min, 85%–25% A; 11–12 min, 25%–2% A; 12–14 min, 2% A; 14–14.1 min, 2%–85% A; 14.1–15 min, 85% A; and 15–16 min, 85% A. A Q Exactive Focus mass spectrometer coupled with Xcalibur software was employed to obtain the MS and MS/MS data based on the IDA acquisition mode. During each acquisition cycle, the mass range was 100–1,500. The top three-parent ions of each cycle were screened, and the corresponding MS/MS data were acquired. The parameters were as follows: sheath gas flow rate, 45 Arb; aux gas flow rate, 15 Arb; capillary temperature, 400°C; full ms resolution, 70,000; MS/MS resolution, 17,500; collision energy, 15/30/45 in NCE mode; and spray voltage, 4.0 kV (positive) or −3.6 kV (negative). Material identification from peaks containing MS/MS data was performed using the secondary mass spectrometry database provided by the Shanghai BIOTREE Biotech Co., Ltd. and the corresponding cleavage law matching method [15].

### 2.3. Analyzing DHHQD Using Network Pharmacology

#### 2.3.1. Screening Active Chemical Ingredients in DHHQD

The chemical ingredients of DHHQD were screened from the TCM systems pharmacology database and analysis platform (https://tcmspw.com/tcmsp.php) and the encyclopedia of traditional Chinese medicine (https://www.tcmip.cn/ETCM) [16], and candidate ingredients with a drug-likeness ≥0.18 and oral bioavailability ≥30% were selected. In addition, PubMed (https://pubmed.ncbi.nlm.nih.gov) was searched for literature related to the use of Dahuang and Huangqi for CKD-RIF to extract the effective components and their roles, which were combined with the identified active components of DHHQD using MS/MS. Further, the corresponding targets of DHHQD from the TCMSP database and SymMap database (https://www.symmap.org) were screened [17].

#### 2.3.2. Screening Potential Targets of RIF

The Online Mendelian Inheritance in Man (OMIM; https://omim.org/) and GeneCards (https://www.genecards.org/) databases were utilized to screen the known RIF-related potential targets. These databases predict human genes and their related diseases. We searched for intersection genes of the RIF and DHHQD target genes.

#### 2.3.3. Constructing the Protein-Protein Interaction (PPI) Network

Network construction was performed as follows: (i) A network between the chemical components of the DHHQD and CKD-RIF targets was constructed using Cytoscape 3.5.1 software, and the core decoction components and intermolecular interactions were analyzed by visualizing networks. (ii) The PPI network of core protein target genes was constructed using the online STRING database (https://string-db.org/). (iii) The topological features of each node in the PPI network were analyzed [18].

#### 2.3.4. Analysis of PPI Network Data

The analysis of the PPI network helps to study the molecular mechanism of a disease and discover new drug targets from a systematic perspective. Here, the PPI network was forecast using the STRING database (https://string-db.org/), and eight typical attributes, such as intersection genes, coexpression, gene fusion events, protein complexes, and genomic neighborhood from curated databases and automated text-mining, of each node were assessed. We retained PPIs with comprehensive scores >0.4, and the remaining parameters were set to the default values in STRING [19].

#### 2.3.5. Bioinformatics Analysis

Gene ontology (GO) and Kyoto encyclopedia of genes and genomes (KEGG) enrichment analyses were performed for the target genes. The GO database was used to classify the differentially expressed genes into biological process (BP), cellular component (CC), and molecular function (MF) categories. Target genes were enriched in KEGG and the 20 most enriched pathways were visualized. Combined with research references [18], the target genes and signaling pathways related to DHHQD in the treatment of RIF were screened to guide animal experimental research.

### 2.4. Animal Experiments to Verify the Therapeutic Effect of DHHQD on RIF

#### 2.4.1. Experimental Animals and DHHQD Administration

Forty male 7-week-old Sprague–Dawley rats (body weight 200 ± 20 g) were obtained from the Laboratory Animal Center of the Chongqing Medical University. All animal experiments were approved by the Animal Experimental Ethics Committee of Chongqing Medical University (Chongqing, China; Animal license No. SCXK:2018-0003) and performed according to the guidelines of the Animal Care Committee of Chongqing Medical University. All rats were housed in a thermostatic-control facility at 22°C with a 12 h light/dark cycle. After 1 week of acclimatization, they were divided randomly into three groups of ten rats each: sham (sham operation rats), model (unilateral ureteral obstruction rats, UUO), DHHQD-H (UUO + DHHQD high-dose-administered rats), and DHHQD-L (UUO + DHHQD low-dose-administered rats) groups. First, the rats in the sham group were anesthetized with an intraperitoneal injection of 2% pentobarbital sodium (30 mg/kg body weight). Second, their abdominal cavities were incised to expose the left ureter. Blunt dissection was performed on the left ureter before the closure of the abdominal cavity using stratified suturing. Apart from the sham group, all other groups underwent the same surgical procedure to establish the UUO model rats. Specifically, after anesthesia with 2% pentobarbital sodium (30 mg/kg body weight), the left ureters of all rats were exposed and bluntly dissected. A double ligature with a 4-0 surgical suture on the upper 1/3 portion of the ureters was applied to block flow through the ureters before closing the abdominal cavities. The DHHQD-H and DHHQD-L group rats were administered 20 mL·kg^−1^·d^−1^ and 10 mL·kg^−1^·d^−1^ DHHQD, respectively, through intragastric gavage for 14 d. The DHHQD-H group dosage was calculated based on body surface area to approximate human equivalence according to previously described methods [20]. The DHHQD-L group rats were administered a half dose. The rats in the sham and model groups received intragastric administration of distilled water (20 mL·kg^−1^·d^−1^) for 14 d. After 2 weeks, all rats were anesthetized with 2% pentobarbital sodium and euthanized. Blood and tissues were harvested from rats that were fasted for 12 h.

#### 2.4.2. Measurement of Biochemical Indices

The blood samples from the rats were centrifuged at 3,500 rpm (1,369.55 × g) for 5 min. The clear supernatant was used for the analysis of SCr and BUN levels using an automatic biochemical analyzer. Subsequently, the renal index of each rat was calculated as the kidney weight/body weight (g/kg). The hydroxyproline (Hyp) content of the kidney was measured using HYP Colorimetric Assay kits (Elabscience, Houston, USA).

#### 2.4.3. Histopathological Analysis of Renal Tissue

Rat renal tissue was first fixed in 4% paraformaldehyde for 48 h, embedded in paraffin, and further sectioned. The 3 *μ*m-thick sections obtained were dewaxed, treated with gradient ethanol, and stained with hematoxylin-eosin (HE), Masson's trichrome, and periodic acid-Schiff (PAS) stains. Pathological analysis of glomeruli and tubules was performed using an Olympus BX53 microscope (Olympus Corporation, Tokyo, Japan).

The interstitial score of the renal tubules was analyzed at a 200× magnification; ten tubules per visual field were observed. According to the range of renal tubular atrophy, tubular type, stromal cell infiltration, and fibrosis, scores from 0 to 3 were assigned as follows: 0 for none; 1 for less than 25%; 2 for 25%–50%; and 3 for 50%–75% [21]. Photo images from each cortex were screened, and scores were added based on tubulointerstitial injury: tubular atrophy, tubular necrosis, and interstitial fibrosis [22, 23].

#### 2.4.4. Electron Microscopy

The morphological and microstructural structures of the kidneys, such as the glomerular basement membrane, mesangial cells, podocytes, endothelial cells, and collagen fibers in the interstitial tissue were examined using transmission electron microscopy (TEM). The renal tissues from the rats were fixed in 2.5% glutaraldehyde and embedded in paraffin. The 70 nm-thick tissue sections were stained and observed using TEM (JEM-1400PLUS, JEOL, Tokyo, Japan).

#### 2.4.5. Immunohistochemistry

The 3 *μ*m-thick renal tissue sections were incubated with citrate antigen retrieval solution for 20 min at 95°C. Thereafter, the sections were stained with a monoclonal antibody against transforming growth factor-*β*1 (TGF-*β*1; Cat# GB13028; dilution 1 : 500; Servicebio, Wuhan, China) and *α*-smooth muscle actin (*α*-SMA; Cat# GB111364; dilution 1 : 500; Servicebio). The sections were incubated with goat antirabbit antibodies overnight and then with a secondary antibody for 50 min. The positive areas were visualized using a DAB Kit (Servicebio). The integrated optical density of protein expression was calculated using ImageJ software (National Institutes of Health, Bethesda, MD, USA).

#### 2.4.6. Enzyme-Linked Immunosorbent Assay

Rat IL-6, epidermal growth factor receptor 2 (EGFR2), vascular endothelial growth factor (VEGF), and eNOS enzyme-linked immunosorbent assay (ELISA) kits (Jonln, Shanghai, China) were used to detect protein levels in the kidney tissues. The protein concentration analysis of each group was performed according to the manufacturer's instructions. The concentrations in each group were compared with Student's *t*-tests after logarithmic transformation.

#### 2.4.7. Real-Time PCR

According to the manufacturers' protocols, total RNA was extracted from renal tissue using TRIzol reagent (Invitrogen, San Diego, CA, USA). Furthermore, the RNA was reverse transcribed into cDNA (Takara Bio Inc., Shiga, Ohtsu, Japan). The PCR cycling conditions were as follows: 95°C for 10 min, followed by 95°C for 15 s and 60°C for 60 s for 40 cycles. Gene expression levels were calculated from the standard curve using the expression of the glyceraldehyde 3-phosphate dehydrogenase (*GAPDH*) gene as a reference. The following primers were used: phosphatidylinositol 3-kinase (PI3K): sense, 5ʹ-AGAGCTTGGAGGACGATGACG-3ʹ, antisense, 5ʹ-TGGACTGGGCTATCTCACTTCG-3ʹ; protein kinase B (AKT): sense, 5ʹ-TCTCAGTGGCACAATGTCAGC-3ʹ, antisense, 5ʹ-TGGGTGAACCTGACCGGAAG-3ʹ; toll-like receptor 4 (TLR4): sense, 5ʹ-AGTTTAGAGAATCTGGTGGCTGTG-3ʹ, antisense, 5ʹ-TTCCCTGAAAGGCTTGGTCT-3ʹ; nuclear factor kappa-B (NF-*κ*B), sense, 5ʹ-GCTCCTTTTCTCAAGCCGATGT-3ʹ, antisense, 5ʹ-CGTAGGTCCTTTTGCGTTTTTC-3ʹ; and GAPDH: forward, 5′-CTGGAGAAACCTGCCAAGTATG-3′, reverse, 5′-GGTGGAAGAATGGGAGTTGCT-3′.

#### 2.4.8. Western Blotting

Renal tissue proteins were extracted, quantified, and visualized using western blotting. First, target proteins were separated by sodium dodecyl sulfate polyacrylamide gel electrophoresis and transferred to polyvinylidene fluoride (PVDF, G6015-0.45, Servicebio) membranes. The PVDF membranes with bound target proteins were then blocked with 5% skim milk for 2 h. Primary antibodies (dilution 1 : 1000) against p-PI3K (BS-5570R, BIOSS, Beijing, China), PI3K (BSM-33219M, BIOSS), p-AKT (AF0908, Affinity, Changzhou, Jiangsu, China), AKT (3063, Cell Signaling Technology, Danvers, MA, USA), TLR4 (GB11519, Servicebio), and NF-*κ*B (ab216409, Abcam, Cambridge, MA, USA) were used, and the membranes were incubated overnight at 4°C on a shaking bed. After washing the membranes, the secondary antibody (1 : 2,000 dilution) was added and incubated at 37°C for 2 h. After applying the ECL color reagent and performing dark chamber exposure imaging, the gray value of the images was analyzed using ImageJ software.

#### 2.4.9. Statistical Analysis

Data analyses were performed using SPSS ver.17.0 (SPSS Inc., Chicago, IL, USA). Data are presented as mean ± standard deviation (SD). Variables in each group were tested to determine if they were normally distributed. One-way analysis of variance (ANOVA) was then performed, followed by a least significant difference (LSD) test or Dunnett's T3 test. Skewed data were presented as median with range or transformed to rank cases for normalization and statistically analyzed. Statistical significance was set at *p* < 0.05.

## 3. Results

### 3.1. Component Analysis of DHHQD

To identify the major chemical components, the DHHQD samples were analyzed using UHPLC-MS/MS. The positive (Figure 1(a)) and negative (Figure 1(b)) ion chromatograms of DHHQD revealed the chemical composition of all compounds. Several components were observed in DHHQD. The identified compounds included epicatechin, quercetin, ginkgolide A, isochlorogenic acid B, biochanin A, glyceryl linoleate, gallic acid, emodin, inermin, cianidanol, afzelin, isoliquiritin, glycitin, formononetin, rhein, and apigenin.

The UHPLC-MS/MS analysis was combined with the TCMSP database. A total of 631 potential pathophysiological targets were collected from the TCMSP database, including frequently studied genes, such as *MAPK*, *NOS*, *MMP*, *STAT*, *PPAR*, *SOD*, *EGFR*, and *IL6*.

### 3.2. Potential Targets of RIF

We obtained 2,490 CKD-RIF-related disease targets from GeneCards and 139 CKD-RIF-related disease targets from OMIM. After removing duplicates, 2,351 disease targets and 197 chemical targets remained. Following the intersection of DHHQD and RIF, we observed 139 common targets. A new Venn diagram was constructed to identify intersection genes between those targeted by the active components of DHHQD and those involved in RIF to identify genes potentially targeted by DHHQD in RIF (Figure 2).

### 3.3. Ingredient Targets Gene-Disease Network

According to the intersection genes of DHHQD and CKD-RIF identified using the Venn diagram, we further constructed a DHHQD components-potential targets-diseases macro network diagram (Figure 3). The network contained 176 nodes (considering the 37 ingredients in DHHQD and 139 ingredient targets) and 615 edges. Rhein, emodin, gallic acid, epicatechin, quercetin, apigenin, and formononetin might have formed the main active ingredients of DHHQD since their content was higher than that of the other ingredients in the UHPLC-MS/MS analysis. Additionally, their analysis demonstrated that they occupied most locations in the network composition.

### 3.4. PPI Network Analysis

To explore the core pharmacological mechanism of DHHQD action against RIF and the antifibrotic properties of DHHQD, we evaluated the core network using topological methods. By analyzing the PPI network, we determined how protein targets interact with each other to exert pharmacological effects. Therefore, we constructed a macro network of DHHQD action against RIF and identified 139 interacting protein targets and 1,775 interactions. The protein target level of each node was equal to the number of edges it was connected to (Figure 4 (a)). The PPI networks of DHHQD and RIF were analyzed statistically. The top 30 core targets were chosen based on the most contacted degree, including protein kinase B alpha, insulin, IL-6, VEGFA, EGFR, mitogen-activated protein kinase 3/8 (MAPK3/8), transcription factor jun (JUN), myelocytomatosis oncogene, EGF, signal transducer and activator of transcription 3, and prostaglandin-endoperoxide synthase 2 (Figure 4 (b)). These proteins may represent key factors involved in the action of DHHQD against RIF.

### 3.5. GO Pathway Enrichment Analysis

The GO pathway analysis includes three aspects, BP, CC, and MF, which were used to analyze the core proteins. In total, there were 1,987 components in BP, 70 in CC, and 144 in MF. The first 20 GO enrichment data items are presented in Figure 5.

Among them, we observed that oxidative stress (GO:0006979), cellular responses to oxidative stress (GO:0034599), and reactive oxygen species (GO:0034614) were closely related to inflammation. Similarly, response to mechanical stimulus (GO:0009612), regulation of apoptotic signaling pathway (GO:2001233), response to radiation (GO:0009314), and cellular response to external stimulus (GO:0071496) were positively related to fibrosis. Most of the targets identified in the PPI analysis were also associated with inflammation (such as MAPK3/8, IL-6, and JUN) and apoptosis (such as AKT, VEGFA, EGFR, and EGF).

### 3.6. KEGG Pathway Enrichment Analysis of DHHQD in the Treatment of RIF

To explore the anti-RIF mechanism of DHHQD, the core proteins were enriched in KEGG analysis. The top 20 signaling pathways were obtained according to the KEGG enrichment analysis results. The results indicated that 131 targets were mapped into 123 KEGG pathways, including the AKT/PI3K signaling pathway, IL-17 signaling pathway, TNF signaling pathway, apoptosis, HIF-1 signaling pathway, EGFR tyrosine kinase inhibitor resistance, and toll-like receptor signaling pathway. Based on analysis of the data and relevant biological processes, the 20 highest significant KEGG signaling pathways were screened out (Figures 6(a) and 6(b)).

The molecular mechanism underlying DHHQD treatment of RIF was further studied. The PI3K-AKT signaling pathway (hsa04151) was the most enriched signaling pathway. Additionally, the most potential core targets were enriched in signaling pathways such as EGFR tyrosine kinase inhibitor resistance (hsa01521), MAPK signaling pathway (hsa04010), ErbB signaling pathway (hsa04012), Ras signaling pathway (hsa04014), HIF-1 signaling pathway (hsa04066), FOXO signaling pathway (hsa04068), toll-like receptor signaling pathway (hsa04620), JAK-STAT signaling pathway (hsa04630), and NF-*κ*B signaling pathway (hsa04064). The data revealed that PI3K-AKT was the most enriched signaling pathway (Figure 6(c)).

Notably, numerous targets such as MAPK, toll-like receptor, NF-*κ*B, FOXO, and JAK-STAT signaling pathway appear in the KEGG analysis, which are directly relevant to the PI3K-AKT signaling pathway [24]. Most of their functions as molecular switches for regulating signaling pathways are involved in inflammation, degradation, cell cycle control, apoptosis [25], and oxidative stress resistance [26]. Consistent with this, fibrosis is scar and tissue sclerosis, which is also caused by chronic inflammatory reactions, oxidative stress reactions, cell cycle control, degradation, and apoptosis [27]. Once the PI3K-AKT signaling pathway becomes active, the activation of various other related signaling pathways, which are involved in apoptosis, protein synthesis, metabolism, and cell cycle, can be accelerated [28]. Consistently, our study supports the assumption that DHHQD could alleviate RIF partly by targeting the PI3K-AKT signaling pathway as well as related signaling pathways, such as the NF-*κ*B and toll-like receptor signaling pathways [29].

### 3.7. Animal Experiments

#### 3.7.1. Administration of DHHQD Ameliorated Renal Function in UUO Rats

The levels of SCr (Figure 7(a)) and BUN (Figure 7(b)) and the renal index (Figure 7(c)) were significantly higher in the UUO groups than in the sham group (*p* < 0.01). Moreover, DHHQD-H and DHHQD-L treatment significantly alleviated the renal changes observed in the untreated UUO rats (*p* < 0.01), and DHHQD-H treatment significantly alleviated the renal changes observed in the DHHQD-L rats (*p* < 0.05). The renal collagen content was assessed by Hyp quantification. The level of Hyp in the renal tissue was significantly increased (*p* < 0.01) in each group compared with that in the sham group, whereas the Hyp content was significantly decreased (*p* < 0.01) in the DHHQD groups compared with that in the UUO group (Figure 7(d)).

#### 3.7.2. Effects of DHHQD on Histopathological Changes and Collagen Deposition

There were no significant histopathological changes in the sham group; in contrast, in the UUO group, we observed increased renal tubular atrophy, edema of renal tubular epithelial cells, cytoplasmic loose light staining, dilation of many renal tubules, local protein tube type, local necrotic cell fragments, diffuse lymphocyte infiltration into interstitial tissue, and inflammatory cell infiltration around local vessels. In the DHHQD-H and DHHQD-L groups, the vascular endothelium was intact, without significant abnormality (Figure 8(a)). Compared with that of the sham group, Masson's trichrome staining of UUO group samples (*p* < 0.01) showed that increased fibrosis was present in the renal interstitium (Figure 8(b)) and that glomerular basement membrane thickening was common (Figure 8(c)). The area ratio of mesangial matrix to glomerular was significantly reduced in the DHHQD-H and DHHQD-L groups compared with that in the UUO group (*p* < 0.01). The area in the DHHQD-H group was also significantly lower than that in the DHHQD-L group (*p* < 0.05; Figure 8(d)). The renal tubular injury and renal fibrosis area, assessed by PAS and Masson's trichrome staining, respectively, were significantly reduced in the DHHQD-H and DHHQD-L groups compared with those in the UUO group (*p* < 0.01). In addition, the renal tubular injury and renal fibrosis area in the DHHQD-H group were significantly lower than those in the DHHQD-L group (*p* < 0.05; Figures 8(e) and 8(f)).

Compared with the untreated UUO group, fewer histopathological changes in renal tissues from the DHHQD-H and DHHQD-L groups were observed. The DHHQD-H and DHHQD-L groups also alleviated the dilatation and atrophy of renal tubules and collagen deposition. The histopathological changes in the DHHQD-H group were slightly improved compared with those in the DHHQD-L group. To further observe the effects of DHHQD-H and DHHQD-L at higher magnification, we performed TEM. The thickness of the glomerular basement membrane was significantly higher in the UUO group than in the sham group, and swelled podocytes, fused foot processes, and mesangial and endothelial cell hyperplasia were observed in the glomerular basement membrane. However, these changes were less pronounced in the DHHQD groups. These findings confirm that our experimental model was successful and indicate that DHHQD administration alleviates the pathological changes and RIF observed in UUO rats. According to these results, DHHQD improves renal function and alleviates the pathological changes, and the effect of high-dose DHHQD was more significant than that of low-dose DHHQD (Figure 9).

#### 3.7.3. Molecular Mechanism of DHHQD Action in Alleviating RIF in UUO Rats

The results of immunohistochemical staining revealed that TGF-*β*1 and *α*-SMA were highly expressed in both the renal interstitium and glomerular epithelial cells of UUO-injured kidneys. The expression of TGF-*β*1 and *α*-SMA was the lowest in the sham group. Notably, TGF-*β*1 (*p* < 0.05) and *α*-SMA (*p* < 0.01) were significantly reduced after DHHQD delivery (Figure 10(a)). The analysis supports that DHHQD-H and DHHQD-L delivery can alleviate TGF-*β*1 and *α*-SMA expression and production in the injured epithelial cells. Furthermore, the protein expression of TGF-*β*1 and *α*-SMA was slightly lower in the DHHQD-H group than in the DHHQD-L group (*p* < 0.05; Figure 10(b)).

Network pharmacology analysis demonstrated that IL-6, EGFR, eNOS, and VEGF were core targets in significant, related fibrosis pathways. Furthermore, the levels of IL-6, EGFR, eNOS, and VEGF in each renal group were detected using ELISA. Compared with those in UUO, DHHQD treatment reduced the levels of IL-6 and EGFR. Simultaneously, DHHQD treatment increased the levels of NOS and VEGF. The results showed that ingestion of DHHQD can attenuate the expression of IL-6 and EGFR in UUO rats and increase the expression of eNOS and VEGF (*p* < 0.05; Figure 11).

We further explored the molecular mechanism through which DHHQD-H affects RIF in UUO rats by performing real-time PCR and western blotting of the core target genes, including PI3K, AKT, TLR4, and NF-*κ*B. DHHQD treatment significantly decreased the mRNA and protein levels of PI3K, AKT, TLR4, and NF-*κ*B (*p* < 0.05) (Figures 12(a)–12(c)).

## 4. Discussion

In TCM, CKD pathogenesis is characterized by Qi deficiency, loss of function, turbidity, and oliguria or anuria, wherein the urinary toxins cannot be excreted, and their levels increase. This condition leads to general symptoms like weakness, dark face, ammonia breath, nausea, and loss of appetite. The main pathophysiological feature of CKD is RIF. Thus, the prevention and treatment of RIF are of great significance for CKD treatment. UUO is an ideal animal model to study RIF, whose pathological manifestations are excessive extracellular matrix (ECM) deposition, causing glomerulosclerosis, hardening, and scarring. RIF is a pathological process that induces an inflammatory reaction, ECM deposition, interstitial scar formation, and stress interaction, resulting in ischemic injury to the nephron's glomerulus. In this process, immune cells migrate into the damaged glomerulus and secrete hypoxia-oxidative stress growth factors, such as TGF-*β*1, which appears to be the grandmaster that elicits numerous signals that culminate in fibrosis and renal parenchymal loss [3]. These growth factors cause the mesangial cells to regress to their immature stem cell state, known as mesangioblasts and secrete ECM. The number of myofibroblasts, characterized by *α*-SMA expression, increases during fibrosis and in turn increases the deposition of ECM and expression of profibrogenic cytokines. Renal fibroblasts are activated under the stimulation of TGF-*β*1, the expression of *α*-SMA in myofibroblasts increases, the activated fibroblasts change their function and phenotype, and the ability to synthesize ECM is further enhanced [30]. This excessive ECM deposition leads to glomerulosclerosis, hardening, and scarring and it diminishes the nephron's ability to filter blood.

RIF is a scar formation process induced by an inflammatory reaction, interstitial scar formation, or hypoxia-oxidative stress interaction. Overexpression of cytokines, renal interstitial cell proliferation disorder, excessive accumulation of ECM, and injury, activation, proliferation, and apoptosis of renal intrinsic cells owing to various reasons ultimately lead to structural deterioration and functional loss in renal tissue [3]. Renal fibrosis presents an uneven focal distribution. The scores for mesangial matrix to glomerular Masson's trichrome staining and PAS staining suggest that DHHQD ameliorates collagen fiber deposition and renal tubular injury significantly in UUO rats. TEM revealed that, in UUO rats, the glomerular basement membrane thickened, the podocytes swelled, and part of the foot process coalesced or overgrew. Pathological and ultrastructural changes in the renal tissue were significantly improved in the DHHQD group compared to those in the untreated UUO group. Cell necrosis and apoptosis cause RIF, which leads to microenvironmental scar formation and the development of renal fibrosis from local lesions [3]. Many collagen fibrils were observed in renal interstitial tissues by TEM. In addition, pathological changes in the glomerulus initially focused on the mesangial matrix and glomerular basement membrane. A previous study has revealed that changes in the ECM are relevant to glomerulosclerosis [31]. The TGF-*β*1 expression levels were previously shown to be high in both the cytoplasm and ECM in scar tissue [32]. Our data revealed that TGF-*β*1 deposition measured via immunohistochemistry in the cytoplasm and nucleus of renal interstitial lesion cells was suppressed in the DHHQD group compared to that in the untreated UUO group. Our results also showed that DHHQD could reduce the pathological changes caused by RIF. Therefore, to establish whether our findings regarding improvement in renal function and pathological changes after DHHQD administration were consistent with our network pharmacology data, we conducted molecular biology experiments on the expression of core genes and proteins observed in the study.

Based on the experience of TCM practitioners, we analyzed the DHHQD prescription using UHPLC-MS/MS and network pharmacology and observed sufficient evidence for the treatment of CKD with the main components of this decoction, such as rhein, emodin, gallic acid, epicatechin, quercetin, apigenin, and formononetin. Previous reports have presented that rhein may decrease interstitial fibrosis through antioxidants via activating the SIRT3/FOXO3a signaling pathway [33]. Research suggests that emodin alleviates kidney dysfunction and tubulointerstitial fibrosis through the modification of gut microbiota disorders and via remarkably reduced IL-6 levels in serum, improved intestinal barrier functions, and downregulated key proteins (TLR4 and NF-*κ*B) expression in the intestinal TLR4 signaling pathway [34]. Peng et al. observed that gallic acid is renal protective in the long-term treatment of CKD via the PI3K/AKT signaling pathway [35]. One study revealed that epicatechin prevented the adverse effects of lipopolysaccharide (LPS) challenge essentially by inhibiting TLR4 upregulation, NOX activation, and consequent downstream events like NF-*κ*B activation [36]. Quercetin alleviates LPS-induced inflammatory responses by upregulation of miR-124 in the human renal tubular epithelial cell line HK-2 [37]. Quercetin also prevents ROS production, reduces the expression of adhesion receptors, and activates the inflammation-related pathways p38MAPK and NF-*κ*B [38]. Apigenin ameliorates hyperuricemic nephropathy by inhibiting renal fibrosis via the Wnt/*β*-catenin pathway [39]. Formononetin provided protective effects by promoting the proliferation of surviving renal tubular cells and inhibiting apoptosis after cisplatin-induced acute kidney injury [40]. However, DHHQD is widely used in clinical practice and is effective in the treatment of CKD [41, 42]. Based on the above analysis of active components contained in DHHQD, the network pharmacology report demonstrated that the pharmacological activities of DHHQD during RIF treatment may predominantly be related to the mechanisms underlying antifibrotic, antiapoptotic, and inflammation-related proteins and signaling pathways. Specifically, IL-6, EGFR, eNOS, and VEGF are the core targets related to the significant fibrosis pathways [43]. Obstructive nephropathy activates the EGFR signaling pathway, which regulates renal cell growth, survival, and proliferation. Overexpression of EGFR could increase the expression and activation of TGF-*β*1 and the release of inflammatory cytokines like IL-6 [44]. IL-6 is a pleiotropic cytokine with a wide range of functions. An increase in IL-6 levels is the main CKD manifestation at the onset of the disease. During acute inflammatory reactions, such as internal trauma, surgery, stress response, and infection, IL-6 is produced rapidly [45]. As an endogenous vasodilator, eNOS can prevent vascular inflammation and thrombosis by inhibiting platelet and leukocyte adhesion [46]. It produces NO and superoxide, which are the strongest known blood vessel dilators. It protects the body from a state of hypoxia and reduces its symptoms [47]. In *in vivo* hypoxia with HIF-1*α* activation, HIF-1*α* can increase VEGF expression through gene regulation, increasing the production of VEGF by the body. After VEGF binds to its receptor, the endothelial cell structure changes, and vascular permeability increases, which eventually causes tissue edema [48]. With the prolongation of operation time in UUO rats, there is a gradual decrease in VEGF expression, which is related to postoperative RIF [49]. VEGF is related to the pathogenesis and progression of angiogenesis-dependent diseases, including inflammatory and diabetes-related diseases. VEGF secreted by renal tubular epithelial cells can activate angiogenesis [50]. Our data also revealed that DHHQD can inhibit the expression of EGFR and IL-6, which simultaneously promotes eNOS and VEGF expression. Regulating these proteins can regulate angiogenesis and hypoxia in the UUO rat kidneys.

Based on our GO enrichment analysis, the critical mechanisms of DHHQD action in RIF include the regulation of apoptosis and anti-inflammatory effects. Combined with KEGG analysis, PI3K/AKT signaling pathways were the most relevant signaling pathways affected by DHHQD in RIF treatment. TLR4, NF-кB, and eNOS are high-frequency research targets, enriched in the TLR4/NF-кB signaling pathway. These signaling pathways lie upstream of the enrichment sequence, wherein the enriched genes with significant *p*values are present. Phosphatidylinositol 3-kinase (PI3K) has Ser/Thr and phosphatidylinositol kinase activities. Tyrosine kinase receptors expressed on the cell surface, such as PDGF receptor and EGFR, bind with their corresponding ligands to activate PI3K, act on phosphatidylinositol 4,5-bisphosphate (PIP2) to generate phosphatidylinositol 3,4,5-trisphosphate (PIP3), bind and activate AKT, and then activate downstream proteins such as CHK1, BAD, FOXO, and other target proteins that regulate cell proliferation and apoptosis. Based on network pharmacology and experimental pharmacology, the PI3K-AKT signaling pathway as a molecular switch for signal pathway regulation is involved in antifibrotic effects, inflammation, oxidative stress resistance, degradation, cell cycle control, and apoptosis [51]. Once the PI3K-AKT signaling pathway is active, the activation of various other related signaling pathways involved in apoptosis, protein synthesis, metabolism, and the cell cycle may also be accelerated [25]. NF-*κ*B exists in the cytoplasm and plays a role in transcription and activation. Under normal conditions, NF-*κ*B and its inhibitor protein I*κ*B are bound and inactive. During inflammation, I*κ*B phosphorylation leads to NF-*κ*B dissociation and activation followed by its translocation to the nucleus, where it promotes ECM generation by modulating gene expression. Previous network pharmacology and experimental pharmacology [52, 53] studies have illustrated that the TLR4/NF-*κ*B or PI3K/AKT signaling pathway can be inhibited by gut microbial-derived metabolites and can exert anti-RIF and anti-inflammatory effects [54, 55]. Here, the mRNAs and proteins of AKT, PI3K, TLR4, and NF-*κ*B in UUO rat kidneys showed reduced expression in response to DHHQD. Therefore, we speculate that DHHQD inhibits PI3K/AKT and TLR4/NF-*κ*B pathway activity and ultimately, inflammation.

## 5. Conclusions

Owing to the complex composition of herbs, this study verified the effectiveness of DHHQD in treating RIF through animal experiments after UHPLC-MS/MS and network pharmacological analysis. However, based on the results of the DHHQD analysis, we intend to conduct animal and cell experiments on the monomer ingredients with high levels or those known to play key roles in the treatment of RIF. Although the initial screening required for such experiments will be a monumental task, it will provide a scientific basis for elucidating the therapeutic effect of DHHQD against RIF and provide new directions for further TCM research and development.

Our network pharmacology analysis and experimental data demonstrated that ingestion of DHHQD can modulate the clinical and pathological changes observed in UUO rats. DHHQD also reduced inflammatory cytokine levels and attenuated collagen deposition, which alleviated renal fibrosis in DHHQD-treated UUO rats. Additionally, the renal protective effect may be related to the downregulation of PI3K/AKT and TLR4/NF-*κ*B pathways; hence, further investigations are warranted.

## Figures and Tables

**Figure 1:** Positive (a) and negative (b) ion chromatograms of Dahuang-Huangqi decoction (DHHQD) demonstrating the chemical composition of all compounds.

**Figure 2:** Venn diagram shows the predicted effects of Dahuang-Huangqi decoction (DHHQD) on renal interstitial fibrosis (RIF). The intersection of DHHQD- and RIF-related targets is illustrated. There were 139 relevant identical targets, most of which are shown.

**Figure 3:** Dahuang-Huangqi decoction (DHHQD)-component-targets network. The network contained 176 nodes (37 DHHQD ingredients and 139 ingredient targets) and 615 edges, which indicated ingredient-target interactions. The yellow arrow nodes represent the bioactive components of DHHQD. The purple square nodes represent the CKD-RIF potential targets. These connections represent the close relationship between the bioactive components in DHHQD and potential targets of CKD-RIF.

**Figure 4:** Dahuang-Huangqi decoction (DHHQD)-renal interstitial fibrosis (RIF) protein-protein interaction (PPI) network of 30 core protein targets. (a) The PPI network. The colored circles represent 139 targets of the protein ingredients of DHHQD, and the lines represent their interactions, which involve 2,615 mechanisms. The more central a circle in the network, the more relevant is the research mechanism. (b) The top 30 core proteins are ranked from bottom to top.

**Figure 5:** Gene ontology (GO) functional analysis. The top 20 significantly enriched GO terms in biological process (BP), cellular component (CC), and molecular function (MF) are presented.

**Figure 6:** Kyoto encyclopedia of genes and genomes (KEGG) pathway enrichment analysis of the Dahuang-Huangqi decoction (DHHQD) and renal interstitial fibrosis (RIF) target-pathway network. KEGG is based on (a) gene ratio and (b) *p*value. (c) The top 20 putative signaling pathways, containing 151 nodes and 7,734 edges. The 131 green nodes represent targets, and the 20 red nodes represent the top 20 KEGG pathways. The edges represent the interactions and node size is proportional to interaction degree.

**Figure 7:** Effects of DHHQD on renal structure/function parameters in UUO rats. (a) Serum creatinine (SCr) and (b) blood urea nitrogen (BUN) levels measured in blood. (c) Renal index and (d) kidney hydroxyproline (Hyp) were also measured (*n* = 10 rats per group). UUO, unilateral ureteral obstruction; DHHQD-H, Dahuang-Huangqi decoction high dose; and DHHQD-L, Dahuang-Huangqi decoction low dose. Data are presented as the mean ± SD. ^*∗*^*p* < 0.05, ^*∗∗*^*p* < 0.1.

**Figure 8:** Histopathology of renal tissue samples. (a) Hematoxylin and eosin (HE) staining presenting high renal tubule atrophy, high tubular epithelial cell edema, cytoplasmic loose light staining (yellow arrow), high renal tubule dilation (green arrow), and diffuse lymphocyte infiltration (blue arrow) into interstitial tissues in unilateral ureteral obstruction (UUO); meanwhile, the pathological changes were mild in the DHHQD-H and DHHQD-L groups. Magnification, 200×. (b) Masson's trichrome staining revealed increased collagen deposition (black arrow) in the UUO rat group and low levels of collagen deposition in the DHHQD-H and DHHQD-L groups; the DHHQD-H group revealed slightly improved collagen deposition compared to that of the DHHQD-L group. Magnification, 200×. (c) Periodic acid-Schiff (PAS) staining presenting glomerular basement membrane thickening (brown arrow); the DHHQD-H and DHHQD-L groups were slightly improved compared with the UUO group, and the DHHQD-H group was slightly improved compared with the DHHQD-L group. Magnification, 200×. (d) The area ratio of mesangial matrix to glomerular in HE staining (%). (e) Tubule injury index score. (f) Collagen volume fraction assessed by Masson's staining (%). DHHQD-H, Dahuang-Huangqi decoction high dose; DHHQD-L, Dahuang-Huangqi decoction low dose. ^*∗*^*p* < 0.05, ^*∗∗*^*p* < 0.1.

**Figure 9:** Effect of Dahuang-Huangqi decoction (DHHQD) as assessed by transmission electron microscopy (TEM) of renal tissue samples (10,000×). (a) The UUO group presented glomerular basement membrane thickening (brown arrow) and mesangial matrix increase, accompanied by extensive podocyte fusion (yellow arrow). These pathological changes were alleviated in the DHHQD-H and DHHQD-L groups. The DHHQD-H group was slightly improved compared with the DHHQD-L group. (b) Collagenous fibers (red arrow) in renal interstitial tissues increased significantly in the UUO group and decreased in the DHHQD-H and DHHQD-L groups. The collagenous fibers were slightly fewer in the DHHQD-H group than in the DHHQD-L group. DHHQD-H, Dahuang-Huangqi decoction high dose; DHHQD-L, Dahuang-Huangqi decoction low dose.

**Figure 10:** Dahuang-Huangqi decoction (DHHQD) treatment minimizes transforming growth factor (TGF)-*β*1 and *α*-smooth muscle actin (*α*-SMA) deposition in the kidneys of unilateral ureteral obstruction (UUO) rats. (a) The protein expression of TGF-*β*1 and *α*-SMA was determined by immunohistochemistry at 400× magnification. Positive staining is brown. (b) The positive area is expressed as the mean percentage ± SD for each experimental group. The protein expression of TGF-*β*1 and *α*-SMA was slightly lower in the DHHQD-H group than in the DHHQD-L group. DHHQD-H, Dahuang-Huangqi decoction high dose; DHHQD-L, Dahuang-Huangqi decoction low dose. ^*∗*^*p* < 0.05, ^*∗∗*^*p* < 0.01.

**Figure 11:** The levels of endothelial nitric oxide synthase (eNOS), epidermal growth factor receptor (EGFR), vascular endothelial growth factor (VEGF), and interleukin (IL)-6 in kidney tissues from individual rats were measured using ELISA. DHHQD treatment reduced the levels of EGFR and IL-6 in UUO rats. DHHQD treatment increased the levels of eNOS and VEGF in UUO rats. Data are presented as the mean ± SD of each group from three separate experiments. DHHQD-H, Dahuang-Huangqi decoction high dose; DHHQD-L, Dahuang-Huangqi decoction low dose; UUO, unilateral ureteral obstruction. ^*∗*^*p* < 0.05, ^*∗∗*^*p* < 0.01.

**Figure 12:** Effects of Dahuang-Huangqi decoction (DHHQD) on PI3K-AKT pathway signaling pathway. Unilateral ureteral obstruction (UUO) rats were administered water or Dahuang-Huangqi decoction (DHHQD) at 20 mL·kg^−1^·d^−1^ by oral gavage for 14 d Sham group rats were administered equal volumes of water. (a) mRNA expression of inflammation-related genes in DHHQD-administered rats compared to that in UUO rats was determined using quantitative reverse transcription-polymerase chain reaction (qRT-PCR) analyses. Glyceraldehyde 3-phosphate dehydrogenase (GAPDH) was used as the internal reference. (b, c) Protein expression levels were determined using western blotting. Data are presented as mean ± SEM. ^*∗*^*p* < 0.05, ^*∗∗*^*p* < 0.01.

## Data Availability

The data that support the findings of this study are available from the corresponding author upon reasonable request.
